The article "CircRNA EPHB4 modulates stem properties and proliferation of gliomas via sponging miR‐637 and up‐regulating SOX10" was retracted in 2024. Reasons: duplicated images; original data or images not available.

# CircRNA EPHB4 modulates stem properties and proliferation of gliomas via sponging miR‐637 and up‐regulating SOX10

**DOI:** 10.1002/1878-0261.12830

**Published:** 2020-12-16

**Authors:** Chen Jin, Jie Zhao, Zhi‐Ping Zhang, Ming Wu, Jian Li, Bo Liu, Xin‐ Bin Liao, Yu‐Xiang Liao, Jing‐Ping Liu

**Affiliations:** ^1^ Department of Neurosurgery Xiangya Hospital Central South University Changsha China

**Keywords:** cancer stemness, circEPHB4, gliomas, miR‐637, proliferation, SOX10

## Abstract

Gliomas are the most common type of primary brain tumors. CircRNA ephrin type‐B receptor 4 (circEPHB4) is a circular RNA derived from the receptor tyrosine kinase EPHB4. However, the clinical significance and the specific roles of circEPHB4 in gliomas and glioma cancer stem cells (CSC) have not been studied. Here, we found that circEPHB4 (hsa_circ_0081519) and SOX10 were up‐regulated and microRNA (miR)‐637 was down‐regulated in glioma tissues and cell lines. Consistently, circEPHB4 was positively correlated with SOX10 but negatively correlated with miR‐637. The altered expressions of these molecules were independently associated with overall survival of patients. CircEPHB4 up‐regulated SOX10 and Nestin by directly sponging miR‐637, thereby stimulating stemness, proliferation and glycolysis of glioma cells. Functionally, silencing circEPHB4 or increasing miR‐637 levels in glioma cells was sufficient to inhibit xenograft growth *in vivo*. In conclusion, the circEPHB4/miR‐637/SOX10/Nestin axis plays a central role in controlling stem properties, self‐renewal and glycolysis of glioma cells and predicts the overall survival of glioma patients. Targeting this axis might provide a therapeutic strategy for malignant gliomas.

## Graphical abstract

Altered expression of circEPHB4, miR‐637 or SOX10 was independently associated with overall survival of glioma patients. By sponging miR‐637, circEPHB4 up‐regulated SOX10 and its target Nestin to promote stemness and self‐proliferation of glioma cells, stimulating the malignant progression of gliomas. Consistently, silencing circEPHB4 or overexpressing miR‐637 inhibited xenograft growth of glioma cells *in vivo* and has therapeutic prospects.

**Abbreviations**
ANOVA: analysis of variance
circEPHB4: circRNA ephrin type‐B receptor 4
circRNA: circular RNA
HK2: hexokinase 2
mRNA: messenger RNA
miRNA: microRNA
PDK1: pyruvate dehydrogenase kinase 1
PI: propidium iodide
PKM2: pyruvate kinase M2
qRT‐PCR: quantitative real‐time polymerase chain reaction
RIP: RNA immunoprecipitation
SD: standard deviation
shcircEPHB4: short hairpin RNA specifically targeting circEPHB4

## 1 Introduction

Gliomas, accounting for approximately 30% of all intracranial tumors, are the most common type of primary brain tumors [1]. Unfortunately, the majority (approximately 80%) of all gliomas are malignant in nature, with a worldwide incidence of 3.9 per 100 000 in males and 3.1 per 100 000 in females [2]. The current treatment options for gliomas are limited to surgery combined with radiotherapy and/or chemotherapy, and have minimal effects on patients with malignant gliomas, leading to a median survival of only 15–16 months for those with stage IV glioblastoma [3]. One molecular mechanism responsible for the aggressive growth, metastasis and therapeutic resistance of malignant gliomas is the presence of cancer stem cells (CSC). CSC are characterized by specific markers such as CD133, CD44, Nestin, Nanog and Oct4, and present biological phenotypes including persistent self‐renewal, active proliferation, and potential for differentiation [4, 5]. Cumulative evidence suggests that CSC play crucial roles in the oncogenesis and recurrence of malignant gliomas [5, 6, 7]. Therefore, elucidating molecular mechanisms regulating cancer stemness of gliomas and developing therapeutics targeting these mechanisms may hold hope for glioma treatment.

Circular RNA (circRNA) are a group of RNA molecules presenting as covalently closed continuous loops and functioning in a variety of biological processes, including encoding peptides [8], acting as sponges for microRNA (miRNA) [9], and regulating gene transcription by sequestering RNA‐binding proteins [10]. As a result, circRNA contribute to the development of many diseases. In cancers, not only are the expression levels of circRNA correlated with distinct clinicopathological characteristics and thus established as cancer biomarkers, but increasing molecular mechanisms have been revealed for their biological functions [11, 12]. The circRNA ephrin type‐B receptor 4 (circEPHB4) is a circRNA derived from the receptor tyrosine kinase EPHB4. Considering the significant, yet dichotomous roles of EPHB4 in human cancers [13], it is speculated that circEPHB4 also critically regulates the development of cancers, as has been demonstrated in hepatocellular carcinoma [14]. A recent study revealed eight highly expressed circRNA, including circEPHB4, in glioma tissues [15]. However, the clinical significance or the specific regulation mechanism underlying circEPHB4 in malignant gliomas, specifically in regulating glioma CSC, has not been studied.

We performed bioinformatic analysis (Circular RNA Interactome) and identified miR‐637, a miRNA characterized as a tumor suppressor in different human cancers [16, 17, 18], as a potential interacting partner for circEPHB4 (hsa_circ_0081519). An earlier study showed that reduced miR‐637 expression was observed in human gliomas, associated with poor prognosis of patients, and promoted glioma growth and invasion via up‐regulating Akt1 [19]. Therefore, we propose that by sponging the tumor suppressor miR‐637 and releasing the suppression of miR‐637 on certain target genes, circEPHB4 might present oncogenic activities. So far, there are no reports on the regulation between circEPHB4 and miR‐637 or the biological importance of this regulation.

In addition to revealing the potential binding sites between circEPBH4 and miR‐637, our preliminary bioinformatic analysis using the RNA Interactome Database showed that SOX10 might bind to miR‐637 at the same sites. SOX10 is a transcription factor that stimulates the CSC feature in breast cancer by up‐regulating Nestin [20, 21]. These clues, combined with reports that SOX10 is highly expressed in gliomas [22, 23] and that reduced miR‐637 expression is an unfavorable prognostic marker for gliomas [19], encouraged us to examine whether miR‐637 might act through SOX10 to regulate stemness of gliomas. This is also the first study to research the interaction between miR‐637 and SOX10.

In this study, we validate a hypothesis that by sponging miR‐637, circEPHB4 (hsa_circ_0081519) up‐regulates SOX10 and Nestin expression to promote the stemness as well as the self‐proliferation of glioma cells. To test this hypothesis, we used both glioma tissues obtained from patients and glioma cell lines, and tested the significance of the circEPHB4/miR‐637/SOX10/Nestin axis *in vitro* and *in vivo*. This is the first study exploring the effects of circEPHB4 on cancer stemness and the first to study the interaction between circEPHB4, miR‐637 and SOX10. Our study suggests that targeting circEPHB4/miR‐637/SOX10 axis benefits glioma therapy.

## 2 Materials and methods

### 2.1 Human samples

This research conforms to the standards set by the Declaration of Helsinki and was approved by the Ethics Committee of Xiangya Hospital, Central South University (Changsha, Hunan, China). All participants gave their written consents. A total of 40 glioma patients were recruited into this study. During the surgery, paired glioma tissues and para‐tumor normal brain tissues were obtained and stored in liquid nitrogen. The clinicopathologic characteristics of these patients are summarized in Table 1.

**Table 1:** Associations between circEPHB4/miR‐637 expression and clinicopathologic characteristics in patients with gliomas

Clinical parameters	Cases (*n*)	Expression level		*P*‐value	Expression level		*P*‐value
		circEPHB4^high^	circEPHB4^low^	(*P < 0.05)	miR‐637^high^	miR‐637^low^	(*P < 0.05)
Age (years)							
≥60	27	16	11	0.1760	10	17	0.0407
<60	13	4	9		10	3	
Gender							
Male	20	2	18	<0.0001	8	12	0.3431
Female	20	18	2		12	8	
Smoking status							
No	14	8	6	0.7411	6	8	0.7411
Yes	26	12	14		14	12	
KPS score							
≤80	25	16	9	0.0484	11	14	0.5145
＞80	15	4	11		9	6	
Tumor location							
Mesenchymal	14	7	7	0.3430	8	6	0.6180
Proneural	12	4	8		5	7	
Classic	8	6	2		5	3	
Neural	6	3	3		2	4	
Tumor subtype							
Astrocytoma	10	6	4	0.0764	5	5	0.7773
Oligodendroglioma	7	6	1		3	4	
Glioblastoma	11	2	9		7	4	
Angiocentric glioma	3	2	1		1	2	
Pilocytic astrocytoma	5	3	2		3	2	
Pleomorphic xanthoastrocytoma	4	1	3		1	3	
WHO grade							
Ⅰ and Ⅱ	18	17	1	<0.0001	4	14	0.0036
Ⅲ and Ⅳ	22	3	19		16	6	
Distant metastasis							
Yes	21	3	18	<0.0001	16	5	0.0012
No	19	17	2		4	15	

### 2.2 Bioinformatic analysis

The correlation analysis between SOX10 and the overall survival of glioma patients was performed using the Jefferson online tool (http://genomics.jefferson.edu/proggene/index.php).

### 2.3 Cell culture, transfection and treatment

The normal human astrocytes NHA and three human glioma cell lines, A172, SHG‐44 and LN229, were purchased from Cell Bank of Shanghai Institute for Biological Sciences (Chinese Academy of Sciences, Shanghai, China) or the American Type Culture Collection (ATCC, Manassas, VA, USA). The cells were cultured in DMEM containing 10% FBS and 100 U·mL^1^ penicillin/streptomycin (all from Gibco, Carlsbad, CA, USA) at 37 °C in a humidified incubator containing 5% CO_2_.

To stably alter circEPHB4 (hsa_circ_0081519), miR‐637 and SOX10 expression levels in glioma cell lines, short hairpin RNA (shRNA) specifically targeting circEPHB4 (shcircEPHB4) and the circEPHB4 sequence for overexpression (OE‐circEPHB4), miR‐637 mimics and inhibitor, or shSOX10 and the SOX10 sequence (OE‐SOX10) were cloned into lentivirus vectors (pCDH‐CMV‐MCS‐EF1‐CopGFP‐T2A‐Puro or pLKO.1‐EGFP‐Puro, GenePharma, Shanghai, China). Lentiviral particles were generated by transfecting lentiviral plasmids into 293T packing cells using the Lenti‐X HTX packaging system (Clontech, San Francisco, CA, USA) according to the manufacturer’s instructions. The resulting lentiviral particles were then transfected into target cells according to the manufacturer’s instructions for 48 h. Then, stable cells were obtained upon culture in puromycin‐containing medium (Invitrogen, Carlsbad, CA, USA) for 10 days. shNC, OE‐NC, mimics NC or inhibitor NC were used in parallel as the corresponding negative controls. The plasmid maps of overexpressing circEPHB4 (hsa_circ_0081519), miR‐637 and SOX10 and the sequences of silencing them are shown in Files S1 and S2, respectively.

### 2.4 Neurosphere formation assay

The neurosphere formation assay was performed as described previously [24]. Briefly, target cells were resuspended in NeuroCult NSC Basal Medium supplemented with growth supplements (all from STEMCELL Technologies, Vancouver, Canada) and seeded into a 35‐mm cell culture dish at 2500 cells per dish. After 21 days, the number of neurospheres with a diameter of ≥ 2 mm was counted under an inverted microscope (Zeiss, Germany).

### 2.5 MTT assay

Cell viability was measured using MTT Assay Kit (Beyotime, Jiangsu, China) according to the manufacturer’s instructions. Briefly, cells growing in log phase were seeded in triplicate at 10^4^ cells·100 μL^‐1^ per well in a 96‐well plate (Corning, Lowell, MA, USA). When treated as indicated, MTT reagent (20 µL per well) was added and incubated with cells at 37 °C for 4 h. Then, the supernatant was discarded and DMSO (150 μL per well) was added. The absorbance was measured using a Bio‐Rad 550 microplate reader (Bio‐Rad, Hercules, CA, USA) at 490 nm.

### 2.6 Colony formation assay

The long‐term proliferation of cells was measured using colony formation assay as described previously [25]. Briefly, cells were seeded into 24‐well plate at 200 cells per well. After incubating the cells at 37 ºC for 10 days, cells were fixed with 100% methanol (Sigma, St. Louis, MO, USA) at room temperature for 10 min followed by staining with 0.5% crystal violet (Sigma) for 5 min. A light microscope (Zeiss, Germany) was used to count the number of cell colonies.

### 2.7 Flow cytometry assay

Flow cytometry was performed on Cytoflex Flow Cytometer (Beckman Coulter, Brea, CA, USA). To measure CD133 expression, cells were washed with PBS and stained with anti‐CD133‐FITC antibody (Thermo Fisher Scientific, Waltham, MA, USA). For cell cycle distribution, cells were fixed in 70% ethanol overnight and then stained with FxCycle™ PI/RNase Staining Solution (Thermo Fisher Scientific) following the manufacturer’s protocol. The percentage (%) of cells with DNA contents representing the G_0_/G_1_, S and G_2_/M phases was analyzed using EXPO32 ADC software (Beckman Coulter). To detect cell apoptosis, cells were stained using the Annexin V‐FITC/propidium iodide (PI) apoptosis detection Kit (Thermo Fisher Scientific) following the manufacturer’s instructions and the percentages (%) of apoptotic cells were reported.

### 2.8 Glucose consumption and lactate production assays

The glucose consumption and the lactate production of target cells were measured using the Glucose Uptake Colorimetric Assay Kit (K676‐100; BioVision, Milpitas, CA, USA) or Lactate Assay Kit (K607‐100; BioVision) respectively following the manufacturer’s protocols.

### 2.9 Luciferase reporter assay

Circular RNA Interactome (https://circinteractome.nia.nih.gov/) and RNA Interactome Database (http://www.rna‐society.org/raid/home.html) were used to predict the miR‐637 binding sites on circEPHB4 (hsa_circ_0081519) and SOX10, respectively. Then, mutations were introduced into the potential binding sequences of SOX10 or circEPHB4. Both the wild‐type and mutant sequences were synthesized by GeneChem (Shanghai, China) and cloned into the pmirGLO vector (Promega, Madison, WI, USA). The reporter vectors were transfected into target cells, together with miR‐637 mimics or miR‐637 inhibitor, or their corresponding negative controls using Lipofectamine 2000 (Invitrogen) according to the manufacturer’s instructions. After 48 h, the luciferase activity was detected using the Dual Luciferase Reporter Assay System (Promega) according to the manufacturer’s instructions.

### 2.10 RNA immunoprecipitation assay

RNA immunoprecipitation (RIP) assay was performed using Imprint RNA Immunoprecipitation Kit (Sigma) following the manufacturer’s instructions. Briefly, cells lysates from LN229 and SHG‐44 cells were incubated with protein A magnetic beads conjugated to either anti‐Ago2 or IgG antibody. The coprecipitated RNA was purified and reversely transcribed into cDNA using PrimeScript RT Master Mix (TaKaRa Bio Inc., Shiga, Japan). The enrichment of circEPHB4 and miR‐637 in the complex pulled down by Ago2 or IgG was detected by qPCR. Target RNA level detected in IgG complex was arbitrally defined as 1.

### 2.11 Xenograft mouse model

The animal protocols were approved by the Institutional Animal Care and Use Committee of Xiangya Hospital, Central South University (Changsha, Hunan, China). Six‐week‐old male BALB/C nude mice were purchased from Shanghai SLAC Laboratory Animal Center (Shanghai, China) and housed in a specific pathogen‐free facility with free access to food and water. On day 0, the mice were randomly divided into four groups (*n* = 5 per group) and target cells (5 × 10^6^ cells per mouse) were subcutaneously injected into the right axillary area. Every 5 days thereafter, a caliper was used to measure the tumor length (L) and width (W), and the tumor volume (V) was calculated as *V* = 0.5 × L × W^2^. On day 30, all mice were euthanized. Xenograft tumors were isolated, weighed and the tumor tissues were further processed for histological and expression analyses.

### 2.12 Immunohistochemistry analysis

Xenograft tumor tissues were fixed in 10% formalin overnight, embedded in paraffin, and cut into 5‐µm‐thick sections. After deparaffinization, the tissue sections were washed with PBS and blocked for endogenous peroxidase activity in 0.3% hydrogen peroxide at room temperature for 10 min, and then blocked for non‐specific binding with PBS containing 5% FBS and 0.3% Triton X‐100 at room temperature for 1 h, followed by the incubation with SOX10 antibody (1 : 200; cat. no. 69661, Cell Signaling Technology, Danvers, MA, USA) at 4 ˚C overnight. After the incubation with the biotinylated anti‐rabbit secondary antibody (1 : 1000; cat. no. ab6720, Abcam, Cambridge, MA, USA) at room temperature for 1 h, the avidin peroxidase conjugate (1 : 2000; cat. no. ab59653, Abcam) was added to tissue sections for 1 h at room temperature. Finally, the target signal was developed using DAB substrate (Vector Labs, Burlingame, CA, USA) and the slides were counterstained with hematoxylin.

### 2.13 Quantitative real‐time polymerase chain reaction

Total RNA from tissues or cells was extracted using Trizol reagent and reverse‐transcribed into cDNA using High‐Capacity cDNA reverse transcription Kit [for messenger RNA (mRNA); Thermo Fisher Scientific] or TaqMan™ MicroRNA Reverse Transcription Kit (for miRNA; Thermo Fisher Scientific) following the manufacturer’s instructions. Quantitative RT‐PCR was performed using Thunderbird SYBR qPCR Kit (TOYOBO, Osaka, Japan) on the StepOnePlus Real‐Time PCR system (Applied Biosystems, Foster City, CA, USA). GAPDH and U6 small nuclear RNA were used as internal references for mRNA and miRNA, respectively. Primers were purchased from Sangon Biotech Co., Ltd. (Shanghai, China). The relative quantification in gene expression was determined using the 2^−ΔΔCt^ method [26].

### 2.14 Western blotting

Tissues or cells were lysed in RIPA buffer containing protease and phosphatase inhibitors (Thermo Fisher Scientific) and measured for protein concentration using the BCA Protein Assay Kit (Sangon Biotech, Shanghai, China). Upon electrophoresis, separated proteins were transferred onto PVDF membrane (Millipore, Billerica, MA, USA), blocked with 5% BSA solution for 1 h at room temperature. The membranes were then incubated with primary antibodies (all from Cell Signaling Technology unless otherwise specified) at 4 °C overnight, including SOX10 (1 : 1000; cat. no. 89356), Nestin (1 : 2000; ab105389; Abcam), Oct4 (1 : 1000; cat. no. 2750), Nanog (1 : 1500; cat. no. 4903), CD133 (1 : 1000; cat. no. 64326), CD44 (1 : 1000; cat. no. 37259), cleaved caspase‐3 (1 : 3000; cat. no. 9664), PARP (1 : 1000; cat. no. 9532), cyclin D1 (1 : 1000; cat. no. 2978), cyclin E1 (1 : 2000; cat. no. 20808), cyclin B1 (1 : 1000; cat. no. 12231), pyruvate kinase M2 (PKM2; 1 : 1000; cat. no. 4053), hexokinase 2 (HK2; 1 : 1000; cat. no. 2867), pyruvate dehydrogenase kinase 1 (PDK1; 1 : 1000; cat. no. 13037) and GAPDH (1 : 5000; cat. no. 5174). Secondary antibody of anti‐rabbit IgG was used in this study (1 : 2000; #ab205718; Abcam). The signal was developed using the ECL substrate (Thermo Fisher Scientific) and analyzed using Quantity One Software (Bio‐Rad).

### 2.15 Statistical analysis

All the experiments were repeated individually at least three times. All data were presented as mean ± standard deviation (SD) and analyzed by SPSS 13.0 software (Chicago, IL, USA). Comparison between two groups was performed using Student’s *t*‐test and comparison between three or more groups using one‐way analysis of variance (ANOVA) followed by Tukey’s post hoc test. The correlation between circEPHB3, SOX10 and miR‐637 was performed using Spearmen correlation analysis. The survival analysis was performed using the Kaplan–Meier method and log‐rank test. The correlation between circEPHB4/miR‐637 expression and clinicopathological characteristics of patients with gliomas was assessed by the Chi‐square test. A *P*‐value < 0.05 was considered statistically significant.

## 3 Results

### 3.1 In glioma tissues or cell lines, CircEPHB4 and SOX10 were up‐regulated, whereas miR‐637 was down‐regulated

Although circEPHB4 was identified as a circRNA up‐regulated in gliomas [15], no study has explored its clinical significance or molecular mechanisms, specifically on regulating CSC. We first profiled the expressions of circEPHB4, miR‐637 and SOX10 in glioma tissues and cell lines. As shown in Fig. 1A, both circEPHB4 and SOX10 were significantly up‐regulated, but miR‐637 was robustly down‐regulated in glioma tissues compared with normal tissues (*n* = 40). When analyzing the relative expression of these three molecules in each individual glioma sample, we found that circEPHB4 expression was up‐regulated in 31 and SOX10 in 25 glioma tissues. However, miR‐637 was down‐regulated in 30 glioma tissues (Fig. 1B). The expression of SOX10 was further randomly examined on the protein level by Western blotting in 20 pairs of glioma tissues and normal tissues, which corroborated its up‐regulation in glioma tissues (Fig. S1). Based on Spearman correlation analysis, there was a negative correlation between circEPHB4 or SOX10 and miR‐637, but a positive correlation between circEPHB4 and SOX10 (Fig. 1C). Kaplan‐‐Meier survival analysis showed that a higher circEPHB4 or SOX10 level was independently correlated with reduced overall survival, whereas a higher miR‐637 was independently correlated with enhanced overall survival of glioma patients (Fig. 1D). As shown in Table 1, high circEPHB4 expression and low miR‐637 expression were associated with advanced clinical stage and distant metastasis. Also, analysis of an independent dataset from The Cancer Genome Atlas (TCGA) revealed the significant correlation between higher SOX10 expression with the reduced overall survival (3 and 5 years) of glioma patients (*n* = 103), and the median survival for patients with high SOX10 expression was 2051 days, shorter than that (2432 days) for patients with low SOX10 expression (Fig. 1E). When compared with NHA cells, we found that the expressions of circEPHB4 and SOX10 were significantly higher and that of miR‐637 lower in all three glioma cell lines (Fig. 1F–H). Since circEPHB4 level was higher in SHG‐44 and LN229 cells than in A172 cells, these two cell lines were used for the subsequent experiments. These data support the prognostic significance of all three molecules in gliomas.

**Fig. 1:** CircEPHB4 and SOX10 were up‐regulated, while miR‐637 was down‐regulated in glioma tissues or cell lines. (A) The expression levels of circEPHB4, miR‐637 and SOX10 were examined by qRT‐PCR in 40 pairs of tumor‐free normal tissues and glioma tissues. (B) The relative expression of circEPHB4, miR‐637 and SOX10 examined in (A) is presented for each individual patient. (C) The correlations between the expression levels of circEPHB4 and miR‐637, circEPHB4 and SOX10, and miR‐637 and SOX10 were analyzed by Spearmen correlation analysis. (D) The correlations between the level of circEPHB4, miR‐637, and SOX10 and the overall survival of glioma patients were analyzed using Kaplan–Meier method. (E) TGCA dataset analyzed by Jefferson online tool (http://genomics.jefferson.edu/proggene/index.php) revealed significant correlation between high SOX10 expression and the reduced overall survival (3 and 5 years) of glioma patients (n = 103). (F,G) SOX10 expression was measured on the protein level by Western blotting and compared between NHA cells and three glioma cell lines A172, SHG‐44 and LN229 cells. (H) The expression levels of circEPHB4, miR‐637 and SOX10 were examined by qRT‐PCR and compared between NHA cells and three glioma cell lines A172, SHG‐44, and LN229. Data are presented as mean ± SD from three independent experiments. Comparison between two groups was performed using Student’s *t*‐test and between three or more groups using one‐way ANOVA followed by Tukey’s post hoc test. *P < 0.05, **P < 0.01 and ***P < 0.001.

### 3.2 CircEPHB4 necessarily and sufficiently promoted cancer stemness of glioma cells

To assess the biological function of circEPHB4 on cancer stemness, circEPHB4 was overexpressed (OE‐circEPHB4) or knocked down (shcircEPHB4) in both LN229 and SHG‐44 cells. As expected, shcircEPHB4 treatment significantly reduced circEPHB4 level (Fig. 2A), whereas OE‐circEPHB4 potently boosted circEPHB4 level (Fig. 2B) in both LN229 and SHG‐44 cells. The neurosphere assay showed that down‐regulating circEPHB4 level significantly reduced the number of neurospheres, whereas up‐regulating its level markedly promoted neurosphere formation (Fig. 2C,D). Corresponding to the effects of circEPHB4 level on neurosphere formation, down‐regulating or up‐regulating circEPHB4 was associated with respectively reduced or increased levels of multiple biomarkers for cancer stemness, including surface expression of CD133 (as detected by flow cytometry; Fig. 2E,F), and cellular levels of Nestin, Oct4, Nanog, CD133 and CD44 (as detected by Western blotting; Fig. 2G,H). These data suggest that circEPHB4 is sufficient to maintain the stemness of glioma cells.

**Fig. 2:** CircEPHB4 necessarily and sufficiently promoted cancer stemness of glioma cells. (A,B) The expression levels of circEPHB4 were measured by qRT‐PCR and compared between indicated cells. (C,D) The stemness of indicated cells was examined by neurosphere formation assay, with representative images of formed neurospheres shown in (C) and the quantification results shown in (D). (E,F) The expression of CD133 on the surface of indicated cells was examined by flow cytometry in (E) and the quantification results are shown in (F). (G,H) The expression levels of stem‐cell markers Nestin, Oct4, Nanog, CD133 and CD44 were measured by Western blotting in indicated cells (G) and quantified as the ratio to GAPDH (H). LN229 or SHG‐44 cells were engineered either to stably knock down (shcircEPHB4) or to overexpress circEPHB4 (OE‐circEPHB4). shNC or OE‐NC vector was used as the corresponding negative control for shcircEPHB4 or OE‐circEPHB4. Data are presented as mean ± SD from three independent experiments. Comparison between two groups was performed using Student’s *t*‐test and between three or more groups using one‐way ANOVA followed by Tukey’s post hoc test. *P < 0.05, **P < 0.01.

### 3.3 CircEPHB4 played a central role in stimulating the viability and proliferation, while inhibiting the apoptosis of glioma cells

In addition to cancer stemness, we also assessed the effects of circEPHB4 on the self‐renewal of glioma cells. As shown in Fig. 3A, knocking down circEPHB4 significantly reduced the cell viability of both LN229 and SHG‐44, whereas overexpressing it dramatically boosted the viability. We then examined the significance of altering circEPHB4 level on long‐term cell proliferation using the colony‐forming assay. Results in Fig. 3B,C showed that shcircEPHB4 treatment was associated with a reduced number of colonies, and OE‐circEPHB4 treatment with an increased number. Cell cycle distribution analysis revealed that reducing endogenous circEPHB4 led to G_1_ arrest, whereas increasing circEPHB4 level stimulated cell cycle progression from G_1_ to S phase (Fig. 3D,E). Furthermore, silencing circEPHB4 promoted apoptosis and overexpressing circEPHB4 reduced apoptosis of both LN229 and SHG‐44 cells (Fig. 3F,G). All changes in phenotypes were reflected on the molecular level, as represented by the up‐regulation of the apoptosis biomarker cleaved caspase‐3 and the down‐regulation of uncleaved PARP, and cyclin D1 and cyclin E1 (proteins stimulated cell cycle progression from G_1_ to S phase) by shcircEPHB4. In the OE‐circEPHB4 treatment group, the reverse regulation of these markers was shown (Fig. 3H,I). In contrast, cyclin B1 was not affected by altering the circEPHB4 level, indicating the specific action of circEPHB4 on G_1_/S transition (Fig. 3H,I). Collectively, besides promoting cell cycle progression and cell proliferation, circEPHB4 inhibits apoptosis and thus improves the self‐renewal of glioma cells.

**Fig. 3:** CircEPHB4 played a central role in stimulating the viability and proliferation of glioma cells, while inhibiting apoptosis. (A) The viability of indicated LN229 or SHG‐44 cells was measured by MTT assay for 1, 2, 3, 4 and 5 days, respectively. (B,C) The long‐term proliferation of indicated cells was examined by colony‐forming assay, with representative images of colonies shown in (B) and the number of colonies in (C). (D,E) The cell‐cycle distribution of indicated cells was measured by staining the cells with PI, followed by flow cytometry. Representative images were presented in (D) and the percentages of cells in different phases of cell cycle presented in (E). (F,G) The apoptosis of indicated cells was measured by co‐staining the cells with Annexin V and PI, followed by flow cytometry. Representative images are presented in (F) and the percentage of Annexin V^+^ apoptotic cells in (G). (H,I) The expression levels of markers for apoptosis, cleaved caspase‐3 and uncleaved PARP, and markers for cell cycle progression, cyclin D1, cyclin E1 and cyclin B1 were examined by Western blotting (H) and quantified as the ratio to GAPDH (I). LN229 or SHG‐44 cells were engineered either to stably knock down (shcircEPHB4) or to overexpress circEPHB4 (OE‐circEPHB4). Short hairpin NC or OE‐NC vector was used as the corresponding negative control for shcircEPHB4 or OE‐circEPHB4. Data are presented as mean ± SD from three independent experiments. Comparison between two groups was performed using Student’s *t*‐test and between three or more groups using one‐way ANOVA followed by Tukey’s post hoc test. *P < 0.05, **P < 0.01 and ***P < 0.001.

### 3.4 MiR‐637 presented biological phenotypes the reverse of those of circEPHB4

Considering that expression levels of circEPHB4 and miR‐637 were negatively associated with each other in glioma tissues (Fig. 1), we next examined the biological effects of miR‐637 in glioma cells. Using miR‐637 mimics and inhibitor, we significantly increased and decreased miR‐637 expression, respectively, in both LN229 and SHG‐44 cells (Fig. 4A,B). In contrast to the phenotypes achieved by altering circEPHB4, elevating miR‐637 level using miR‐637 mimics inhibited neurosphere formation (Fig. 4C,D) and down‐regulated cell surface expression of CD133 (Fig. 4E,F), as well as the expression of multiple stemness biomarkers, including Nestin, Oct4, Nanog, CD133 and CD44 (Fig. 4G,H). In contrast, miR‐637 inhibitor presented opposite effects in regulating stemness features of glioma cells (Fig. 4C–H).

**Fig. 4:** MiR‐637 displayed stemness‐related phenotypes that were opposite those displayed by circEPHB4. (A,B) The expression of miR‐637 was examined by qRT‐PCR and compared between indicated cells. (C,D) The stemness of indicated cells was examined by neurosphere formation assay, with representative images of formed neurospheres shown in (C) and the quantification results in (D). (E,F) The expression of CD133 on the surface of indicated cells was examined by flow cytometry in (E) and the quantification results shown in (F). (G,H) The expression levels of stem‐cell markers Nestin, Oct4, Nanog, CD133 and CD44 were measured by Western blotting in indicated cells (G) and quantified as the ratio to GAPDH (H). MiR‐637 mimics or miR‐637 inhibitor was transfected into LN229 or SHG‐44 cells to either overexpress or knockdown miR‐637. Data are presented as mean ± SD from three independent experiments. Comparison between two groups was performed using Student’s *t*‐test and between three or more groups using one‐way ANOVA followed by Tukey’s post hoc test. *P < 0.05, **P < 0.01.

Besides the regulation on stemness, miR‐637 mimics suppressed cell viability (Fig. 5A), colony formation (Fig. 5B,C) and cell cycle progression through the G_1_ to S transition (Fig. 5D,E), but promoted apoptosis (Fig. 5F,G). Again, targeting endogenous miR‐637 using miR‐637 inhibitor presented opposite phenotypes (Fig. 5A–G). Mechanistically, we observed the necessary and sufficient role of miR‐637 in regulating cleaved caspase‐3, uncleaved PARP, cyclin D1 and cyclin E1, but not cyclin B1 (Fig. 5H,I), the reverse of the regulation conferred by circEPHB4. Therefore, miR‐637 demonstrates essential anti‐tumor activities, including inhibiting stem properties and suppressing the proliferation of glioma cells.

**Fig. 5:** MiR‐637 displayed proliferation‐related phenotypes opposite to those displayed by circEPHB4. (A) The viability of indicated LN229 or SHG‐44 cells was measured by MTT assay for 1, 2, 3, 4 and 5 days, respectively. (B,C) The long‐term proliferation of indicated cells was examined by colony‐forming assay, with representative images of colonies shown in (B) and the number of colonies in (C). (D,E) The cell‐cycle distribution of indicated cells was measured by staining the cells with PI, followed by flow cytometry. Representative images were presented in (D) and the percentages of cells in different phases of cell cycle in (E). (F,G) The apoptosis of indicated cells was measured by co‐staining the cells with Annexin V and PI, followed by flow cytometry. Representative images were presented in (F) and the percentage of Annexin V^+^ apoptotic cells in (G). (H,I) The expression levels of markers for apoptosis, cleaved caspase‐3 and uncleaved PARP, and markers for cell cycle progression, cyclin D1, cyclin E1 and cyclin B1, were examined by Western blotting (H) and quantified as the ratio to GAPDH (I). MiR‐637 mimics or miR‐637 inhibitor was transfected into LN229 or SHG‐44 cells to either overexpress or knockdown miR‐637. Data are presented as mean ± SD from three independent experiments. Comparison between two groups was performed using Student’s *t*‐test and between three or more groups using one‐way ANOVA followed by Tukey’s post hoc test. *P < 0.05, **P < 0.01 and ***P < 0.001.

### 3.5 CircEPHB4 directly targeted the expression of miR‐637

One mechanism for circRNA is by binding to miRNA and functioning as miRNA sponges, thus suppressing miRNA functions [27]. To examine whether circEPHB4 functions as a sponge for miR‐637, we first measured the expression of miR‐637 after circEPHB4 overexpression or knocking down. As shown in Fig. 6A,B, the level of miR‐637 was significantly boosted in shcircEPHB4 cells but potently reduced in OE‐circEPHB4 cells. Sequence analysis revealed the potential binding site within circEPHB4 to miR‐637 (Fig. 6C). We then found that miR‐637 mimics and inhibitor only, specifically inhibited and promoted the luciferase activity driven by wild‐type sequences, respectively, but did not alter the luciferase activity driven by mutated sequences (Fig. 6D). The endogenous interaction between circEPHB4 and miR‐637 was further corroborated by RIP assay, where in both LN229 and SHG‐44 cells, circEPHB4 and miR‐637 were significantly enriched in Ago2‐containing complex (Fig. 6E), suggesting that circEPHB4 directly binds to miR‐637 and thus may function as a sponge for miR‐637.

**Fig. 6:** CircEPHB4 directly targeted the expression of miR‐637. (A,B) The expression of miR‐637 was measured by qRT‐PCR in LN229 or SHG‐44 cells with altered expression of circEPHB4. (C) Bioinformatic analysis revealed a potential binding site between circEPHB4 and miR‐637. (D) The luciferase activity was measured by reporter assay. Wild‐type (WT) or mutated (MUT) circEPHB4 sequence was cloned into luciferase reporter construct, co‐transfected into LN229 or SHG‐44 cells with either miR‐637 mimics or inhibitor. (E) The interaction between circEPHB4 and miR‐637 was examined by RIP assay using either anti‐Ago2 or IgG antibody. The level of circEPHB4 or miR‐637 pulled down by IgG was arbitrally defined as 1. Data are presented as mean ± SD from three independent experiments. Comparison between two groups was performed using Student’s *t*‐test and between three or more groups using one‐way ANOVA followed by Tukey’s post hoc test. *P < 0.05, **P < 0.01.

### 3.6 MiR‐637 antagonized myriad biological effects of circEPHB4 in glioma cells

To assess the significance of miR‐637 in the biological activities of circEPHB4, we treated shcircEPHB4 cells (LN229) with miR‐637 inhibitor. As shown in Fig. 7A, miR‐637 inhibitor significantly reduced endogenous miR‐637 level caused by shcircEPHB4. Corresponding to the reduction in miR‐637, we observed increases in cell viability (Fig. 7B) and neurosphere formation (Fig. 7C,D) and up‐regulation of cell‐surface CD133 (Fig. 7E,F) as well as other stemness biomarkers (Fig. 7G,H), all of which were effected by shcircEPHB4.

**Fig. 7:** Knocking down miR‐637 reversed anti‐stemness phenotypes conferred by shcircEPHB4. (A) The expression of miR‐637 was measured by qRT‐PCR in indicated LN229 cells. (B) The viability of indicated LN229 cells was measured by MTT assay for 1, 2, 3, 4 and 5 days, respectively. (C,D) The stemness of indicated cells was examined by neurosphere formation assay, with representative images of formed neurospheres shown in (C) and the quantification results in (D). (E,F) The expression of CD133 on the surface of indicated cells was examined by flow cytometry in (E) and the quantification results are shown in (F). (G,H) The expression levels of the stem‐cell markers Nestin, Oct4, Nanog, CD133 and CD44 were measured by Western blot in indicated cells (G) and quantified as the ratio to GAPDH (H). LN229 cells were simultaneously manipulated for the levels of circEPHB4 and miR‐637 (shcircEPHB4 + miR‐637 inhibitor). Data are presented as mean ± SD from three independent experiments. Comparison between three or more groups was performed using one‐way ANOVA followed by Tukey’s post hoc test. *P < 0.05, **P < 0.01 and ***P < 0.001.

We also detected enhanced colony formation (Fig. 8A,B), G_1_/S transition (Fig. 8C,D), suppression of cell apoptosis (Fig. 8E,F) and cleaved caspase‐3, and increase in uncleaved PARP, cyclin D1 and cyclin E1 (Fig. 8G,H) by the miR‐637 inhibitor when compared with cells with shcircEPHB4 treatment alone.

**Fig. 8:** Knocking down miR‐637 reversed anti‐proliferation phenotypes conferred by shcircEPHB4. (A,B) The long‐term proliferation of indicated cells was examined by colony‐forming assay, with representative images of colonies shown in (A) and the number of colonies in (B). (C,D) The cell‐cycle distribution of indicated cells was measured by staining the cells with PI, followed by flow cytometry. Representative images were presented in (C) and the percentages of cells in different phases of cell cycle are presented in (D). (E,F) The apoptosis of indicated cells was measured by co‐staining the cells with Annexin V and PI, followed by flow cytometry. Representative images were presented in (E) and the percentage of Annexin V^+^ apoptotic cells in (F). (G,H) The expression levels of markers for apoptosis, cleaved caspase‐3 and uncleaved PARP, and markers for cell cycle progression, cyclin D1, cyclin E1 and cyclin B1, were examined by Western blotting (G), and quantified as the ratio to GAPDH (H). (I,J) Glucose consumption (I) and lactate production (J) from indicated cells were measured using corresponding assay kits. (K,L) The expression levels of glycolysis‐related biomarkers PKM2, HK2, and PDK1 were examined by Western blotting (K), and quantified as the ratio to β‐tubulin (L). LN229 cells were simultaneously manipulated for the levels of circEPHB4 and miR‐637 (shcircEPHB4 + miR‐637 inhibitor). Data are presented as mean ± SD from three independent experiments. Comparison between three or more groups was performed using one‐way ANOVA followed by Tukey’s post hoc test. *P < 0.05, **P < 0.01 and ***P < 0.001.

Lastly, since cancer cells need to rewire their metabolism and preferentially use glycolysis to support their malignant growth and metastasis [28], we examined the impacts of circEPHB4 and miR‐637 on glycolysis. We found that knocking down circEPHB4 alone was sufficient to reduce glucose consumption (Fig. 8I), lactate production (Fig. 8J) and expression levels of glycolysis‐related biomarkers, including PKM2, HK2 and PDK1 (Fig. 8K,L). All these glycolysis‐inhibitory effects of shcircEPHB4 were rescued by miR‐637 inhibitor (Fig. 8I–L). Our data suggest that miR‐637 acts downstream of circEPHB4 and reverses the pro‐tumor effects of circEPHB4 in glioma cells.

### 3.7 SOX10 was a direct target of miR‐637 in glioma cells

To explore the molecular targets of miR‐637 that may convey its control of multiple malignant phenotypes in glioma cells, we found that miR‐637 mimics were sufficient to reduce SOX10 expression, whereas miR‐637 inhibitor did the opposite on both mRNA (Fig. 9A,B) and protein (Fig. 9C,D) levels. Bioinformatic analysis was performed and identified SOX10 as a potential target for miR‐637 (Fig. 9E). As indicated in Fig. 9F, miR‐637 mimics significantly suppressed, whereas miR‐647 inhibitor potently boosted the luciferase activity driven by wild‐type sequences but not by mutated sequences, indicating that SOX10 is a direct target of miR‐637.

**Fig. 9:** SOX10 was a direct target for miR‐637 in glioma cells. (A–D) The expression levels of SOX10 were measured by qRT‐PCR (A,B) or by Western blotting (C,D) in LN229 or SHG‐44 cells treated with miR‐637 mimics or inhibitor. (E) Bioinformatic analysis identified a potential binding site between miR‐637 and the 3’‐UTR sequences of SOX10. (F) The luciferase activity was measured by reporter assay. Wild‐type (WT) or mutated (MUT) SOX10 binding sequence was cloned into the reporter construct, co‐transfected into LN229 or SHG‐44 cells with either miR‐637 mimics or inhibitor. Data are presented as mean ± SD from three independent experiments. Comparison between two groups was performed using Student’s *t*‐test and between three or more groups using one‐way ANOVA followed by Tukey’s post hoc test. *P < 0.05, **P < 0.01.

### 3.8 Overexpression of SOX10 antagonized the anti‐cancer activities of miR‐637

To address the importance of targeting SOX10 in the biological activities of miR‐637 in glioma cells, we overexpressed SOX10 (OE‐SOX10) in LN229 cells treated with and without miR‐637 mimics. Although overexpressing SOX10 did not alter the endogenous miR‐637 level (Fig. 10A), it did elevate SOX10 mRNA (Fig. 10B) and protein (Fig. 10C,D) levels robustly. What’s more, overexpressing SOX10 reversed SOX10 mRNA (Fig. 10B) and protein (Fig. 10C,D) levels induced by the miR‐637 mimics. Functionally, miR‐637 mimics presented the lower capability to form neurospheres (Fig. 10E,F) and decreased expression levels of multiple stemness markers, including CD133, Nestin, Oct4, Nanog and CD44 (Fig. 10G–J); overexpressing SOX10 alone had the opposite effect. Furthermore, overexpressing miR‐637 together with SOX10 negated the effects of each alone **(**Fig. 10E–J).

**Fig. 10:** SOX10 overexpression rescued the anti‐stemness phenotypes caused by miR‐637. (A) The expression of miR‐637 was measured by qRT‐PCR in indicated LN229 cells. (B) The expression of SOX10 was measured by qRT‐PCR in indicated LN229 cells. (C,D) The expression of SOX10 was measured by Western blotting in indicated LN229 cells. (E,F) The stemness of indicated cells was examined by neurosphere formation assay, with representative images of formed neurospheres shown in (E) and the quantification results in (F). (G,H) The expression of CD133 on the surface of indicated cells was examined by flow cytometry in (G) and the quantification results are shown in (H). (I,J) The expression levels of stem‐cell markers Nestin, Oct4, Nanog, CD133 and CD44 were measured by Western blotting in indicated cells (I) and are quantified as the ratio to GAPDH (J). (K) The viability of indicated LN229 cells was measured by MTT assay for 1, 2, 3, 4 and 5 days, respectively. LN229 cells were overexpressed miR‐637 (miR‐637 mimics), SOX10 (OE‐SOX10) or both (miR‐637 mimics + OE‐SOX10). Data are presented as mean ± SD from three independent experiments. Comparison between three or more groups was performed using one‐way ANOVA followed by Tukey’s post hoc test. *P < 0.05, **P < 0.01 and ***P < 0.001.

In addition to impacting stem cell features, overexpressing SOX10 alone in glioma cells also stimulated cell viability (Fig. 10K), colony formation (Fig. 11A,B) and cell cycle progression from G_1_ to S phase (Fig. 11C,D), while suppressing apoptosis (Fig. 11E,F), whereas treating the same cells with miR‐637 mimics alone, presented opposite phenotypes. Simultaneous overexpression of miR‐637 and SOX10 abolished their individual effects (Figs 10K and 11A–F). These changes were associated with reduced cleaved caspase‐3 and increased uncleaved PARP, cyclin D1 and cyclin E1 after SOX10 overexpression (Fig. 11G,H). Furthermore, miR‐637 mimics and SOX10 had opposite effects on the regulation of glycolysis, the former markedly reducing and the latter significantly promoting glucose consumption (Fig. 11I), lactate production (Fig. 11J) and expression levels of PKM2, HK2 and PDK1 (Fig. 11K,L). Similarly, overexpression of SOX10 partly abolished the impacts of miR‐637 on glycolysis (Fig. 11I–L).

**Fig. 11:** SOX10 overexpression rescued the anti‐proliferation phenotypes caused by miR‐637. (A,B) The long‐term proliferation of indicated LN229 cells was examined by colony‐forming assay, with representative images of colonies shown in (A) and the number of colonies in (B). (C,D) The cell‐cycle distribution of indicated cells was measured by staining the cells with PI, followed by flow cytometry. Representative images were presented in (C) and the percentages of cells in different phases of cell cycle in (D). (E,F) The apoptosis of indicated cells was measured by co‐staining the cells with Annexin V and PI, followed by flow cytometry. Representative images were presented in (E) and the percentage of Annexin V^+^ apoptotic cells in (F). (G,H) The expression levels of markers for apoptosis, cleaved caspase‐3 and uncleaved PARP, and markers for cell cycle progression, cyclin D1, cyclin E1 and cyclin B1, were examined by Western blotting (G) and quantified as the ratio to GAPDH (H). (I,J) Glucose consumption (I) and lactate production (J) from indicated cells were measured using corresponding assay kits. (K,L) The expression of glycolysis‐related biomarkers PKM2, HK2 and PDK1 were examined by Western blotting (K) and quantified as the ratio to β‐tubulin (L). LN229 cells were overexpressed miR‐637 (miR‐637 mimics), SOX10 (OE‐SOX10) or both (miR‐637 mimics + OE‐SOX10). Data are presented as mean ± SD from three independent experiments. Comparison between three or more groups was performed using one‐way ANOVA followed by Tukey’s post hoc test. *P < 0.05, **P < 0.01 and ***P < 0.001.

### 3.9 Knocking down SOX10 had the reverse effect on phenotypes as silencing miR‐637 did

Besides the gain‐of‐function approach, we also applied the loss‐of‐function strategy and knocked down miR‐637 and SOX10 levels in LN229 cells. shSOX10 and miR‐637 inhibitor acted in opposite ways; knocking down SOX10 alone, suppressed the neurosphere formation (Fig. 12A,B), down‐regulating the expression of CD133, Nestin, Oct4, Nanog, and CD44 (Fig. 12C–F), and inhibiting colony formation (Fig. 13A,B) and cell cycle progression from the G_1_ to S phase (Fig. 13C,D), while promoting cell apoptosis (Fig. 13E,F). Silencing SOX10 alone also increased cleaved caspase‐3 and decreased uncleaved PARP, cyclin D1 and cyclin E1 (Fig. 13G,H). Again, knocking down SOX10 partly cancelled the effects caused by miR‐637 inhibitor (Figs 12 and 13). These data imply that SOX10 is a key downstream target of miR‐637 and that suppression of SOX10 is a mechanism accounting for the anti‐cancer activities of miR‐637.

**Fig. 12:** Knocking down SOX10 antagonized the pro‐stemness phenotypes induced by miR‐637 inhibitor. (A,B) The stemness of indicated LN229 cells was examined by neurosphere formation assay, with representative images of formed neurospheres shown in (A) and the quantification results in (B). (C,D) The expression of CD133 on the surface of indicated cells was examined by flow cytometry in (C) and the quantification results are shown in (D). (E,F) The expression levels of stem‐cell markers Nestin, Oct4, Nanog, CD133 and CD44 were measured by Western blotting in indicated cells (E) and quantified as the ratio to GAPDH (F). Data are presented as mean ± SD from three independent experiments. Comparison between three or more groups was performed using one‐way ANOVA followed by Tukey’s post hoc test. *P < 0.05, **P < 0.01 and ***P < 0.001.

**Fig. 13:** Knocking down SOX10 abolished the pro‐proliferation phenotypes conferred by miR‐637 inhibitor. (A,B) The long‐term proliferation of indicated LN229 cells was examined by colony‐forming assay, with representative images of colonies shown in (A) and the number of colonies in (B). (C,D) The cell‐cycle distribution of indicated cells was measured by staining the cells with PI, followed by flow cytometry. Representative images are presented in (C) and the percentages of cells in different phases of cell cycle in (D). (E,F) The apoptosis of indicated cells was measured by co‐staining the cells with Annexin V and PI, followed by flow cytometry. Representative images are presented in (E) and the percentage of Annexin V^+^ apoptotic cells in (F). (G,H) The expression levels of markers for apoptosis, cleaved caspase‐3 and uncleaved PARP, and markers for cell cycle progression, cyclin D1, cyclin E1 and cyclin B1, were examined by Western blotting (G) and quantified as the ratio to GAPDH (H). Data are presented as mean ± SD from three independent experiments. Comparison between three or more groups was performed using one‐way ANOVA followed by Tukey’s post hoc test. *P < 0.05, **P < 0.01 and ***P < 0.001.

### 3.10 Knocking down circEPHB4 or up‐regulating miR‐637 inhibited the *in vivo* xenograft growth of glioma cells

To test whether the above *in vitro* phenotypes may also translate *in vivo*, we established xenografts using LN229 or SHG‐44 cells expressing shcircEPHB4 or miR‐637 mimics. As shown in Fig. 14A–C, both shcircEPHB4 and miR‐637 mimics significantly inhibited *in vivo* xenograft growth as shown by tumor weight and volume, when compared with shNC and NC mimics cells, respectively. When measuring xenograft tumors for gene expressions, we found down‐regulation of circEPHB4, SOX10 and Nestin but up‐regulation of miR‐637 in shcircEPHB4 xenografts (Fig. 14D,F,G). Similarly, overexpressing miR‐637 in xenografts also significantly reduced both SOX10 and Nestin in mRNA and protein levels (Fig. 14E–G). Further immunohistochemical analysis of xenograft tumors showed that xenografts derived from shcircEPHB4 or miR‐637 mimics cells presented a significant reduction of SOX10 protein (Fig. 14H). These results imply that knocking down circEPHB4 or overexpressing miR‐637 inhibits glioma growth *in vivo*, which is associated with the targeting of cancer stemness.

**Fig. 14:** Knocking down circEPHB4 or up‐regulating miR‐637 inhibited the *in vivo* xenograft growth of glioma cells. (A) Images of xenograft tumors from indicated groups. (B) Weights of all xenograft tumors were measured and compared between indicated groups. (C) The growth curve of xenograft tumors is presented as changes in tumor volumes from indicated groups. (D) The expression levels of circEPHB4, miR‐637, SOX10 and Nestin were examined by qRT‐PCR in xenograft tumors derived from indicated cells. (E) The expression levels of miR‐637, SOX10 and Nestin were examined by qRT‐PCR in xenograft tumors derived from indicated cells. (F,G) The expression levels of SOX10 and Nestin were examined by Western blotting in xenograft tumors derived from indicated cells. The representative images are shown in (F) and quantified as the ratio to GAPDH (G). (H) Histological analysis on SOX10 from indicated xenograft tumors. Scale bar: 50 µm. LN229 or SHG‐44 cells expressing shcircEPHB4 or miR‐637 mimics were subcutaneously injected into nude mice (*n* = 5/group). After 30 days, all mice were euthanized. Data are presented as mean ± SD from three independent experiments. Comparison between two groups was performed using Student’s *t*‐test and between three or more groups using one‐way ANOVA followed by Tukey’s post hoc test. *P < 0.05, **P < 0.01.

## 4 Discussion

In this study, we identified for the first time the signaling cascade circEPHB4/miR‐637/SOX10/Nestin as the crucial regulator of glioma stemness and proliferation. By sponging miR‐637 and thus releasing its suppression on SOX10, circEPHB4 stimulated the stemness properties as well as the self‐proliferation of glioma cells. Consequently, targeting circEPHB4 and SOX10 or boosting miR‐637 ameliorated xenograft growth of glioma cells and might therefore become therapeutic strategy for malignant gliomas.

Although circRNA were first discovered in 1976 [29], they did not receive any attention until Salzman *et al*. suggested that these molecules were functional transcript isoforms of human genes [30]. Since then, studies on circRNA have revealed not only their action mechanisms but also their functional significance in different physiological and pathological paradigms, including gliomas. For example, circNT5E and circNFIX promoted proliferation, migration and invasion of glioma cells but inhibited apoptosis [31, 32]. CircITCH inhibited glioma proliferation [33], and both circZNF292 and circSHKBP1 regulated blood vessel formation of gliomas [34, 35]. Although extensive studies assessed the effects of the receptor tyrosine kinase EPHB4, which presented paradoxical activities during cancer development [36], few looked into the involvement of circEPHB4 in human cancers. Tan *et al*. reported that circEPHB4 was down‐regulated in hepatocellular carcinoma, negatively correlated with tumor weight, size and metastasis in a mouse model, and inhibited viability, migration and invasion but induced apoptosis,[14] supporting circEPHB4 as a tumor suppressor in hepatocellular carcinoma. In contrast, Song *et al*. [15] identified circEPHB4 as one of the most significantly up‐regulated circRNA in gliomas, supporting its oncogenic activities. Consistently, we show here that not only was the expression of circEPHB4 up‐regulated in glioma tissues or cell lines and its level correlated with a poorer overall prognosis of glioma patients, it also essentially contributed to the stem‐cell properties (as demonstrated by neurosphere formation and expression profiles of distinct CSC biomarkers), active proliferation (as illustrated by cell viability, colony formation, cell‐cycle distribution, apoptosis and expressional analysis of apoptosis‐ and proliferation‐related biomarkers) and glycolysis (as revealed by glucose consumption, lactate production and expressional analysis of glycolysis‐related biomarkers) of glioma cells *in vitro*. Furthermore, silencing of circEPHB4 inhibited xenograft growth *in vivo*. This is the first study to reveal the clinical significance and detailed regulatory functions of circEPHB4 in malignant gliomas, specifically its effects on glycolysis, demonstrating its importance as a promising prognosis biomarker as well as a therapeutic target for gliomas.

Several mechanisms were revealed for the biological functions of circRNA, including acting primarily as miRNA sponges, regulating RNA transcription via direct binding to DNA locus or RNA polymerase II, serving as a miRNA reservoir, and sequestering RNA‐binding proteins [11, 37]. Via bioinformatic analysis, we identified miR‐637 as a potential interacting partner of circEPHB4. With respect to its clinical significance, miR‐637 was down‐regulated in glioma tissues and its reduced level was associated with poor prognosis of glioma patients. Functionally, we showed that miR‐637 was both necessary and sufficient in inhibiting cancer stemness, proliferation and glycolysis of glioma cells, while promoting apoptosis. *In vivo*, overexpressing miR‐637, similar to knocking down circEPHB4, inhibited xenograft growth. Therefore, miR‐637 presented the opposite functional phenotypes to circEPHB4, which was further corroborated by the reverse expressional correlation between these two RNA molecules in glioma tissues. We also proved for the first time that circEPHB4 directly and negatively regulated miR‐637 expression via luciferase reporter and RIP assays. Furthermore, reducing the miR‐637 level was sufficient to reverse shcircEPHB4‐induced phenotypes. Studies in other cancers have established miR‐637 as a consistent tumor suppressor [16, 17, 18]. In gliomas, Que *et al*. showed that reduced miR‐637 level was an unfavorable prognosis biomarker, and miR‐637 inhibited the proliferation, migration and invasion of glioma cells by direct targeting of Akt1 [19]. Here, we added stemness‐regulation to the functional repertoire of miR‐637. What’s more, we are the first to study the interaction between circEPHB4 and miR‐637. In this study, while knocking down or overexpressing circEPHB4 and miR‐637 did not lead to robust changes (less than threefold) of these target molecules, our repeated *in vitro* experiments revealed that the functional phenotypes caused by these moderate changes were statistically and biologically significant (Figs 2, 3, 4, 5), supporting their significance in gliomas.

In addition to the negative correlation between circEPHB4 and miR‐637 in gliomas, we also revealed a positive correlation between circEPHB4 and SOX10, as well as a negative correlation between miR‐637 and SOX10. SOX10 is a key transcription factor for oligodendroglial differentiation and is ubiquitously expressed in gliomas [22, 23]. Although it was well established that SOX10 stimulated stem cell properties of breast cancer [20, 21], little is known about its involvement in glioma stemness. In this study, we showed for the first time that higher SOX10 level was associated with poor survival of glioma patients and that SOX10 was a direct downstream target of miR‐637. Overexpressing SOX10 alone potently promoted cancer stemness, proliferation and glycolytic phenotypes of glioma cells, whereas knocking down SOX10 inhibited these phenotypes. Furthermore, overexpressing SOX10 sufficiently reversed the inhibition of the above phenotypes presented by overexpressing miR‐637, whereas knocking down SOX10 antagonized the phenotypes induced by silencing miR‐637. Feng *et al*. showed that SOX10 directly activated the transcription of Nestin and thus promoted the cancer stem‐cell properties of triple‐negative breast cancer cells [21]. Here, we also showed that SOX10 was able to abolish the inhibition of miR‐637 on Nestin expression, supporting that maintaining Nestin expression was at least one mechanism by which SOX10 promoted cancer stemness in glioma cells. Considering that Akt1 was also demonstrated to be a target of miR‐637 [19], it will be interesting to examine the crosstalk between Akt1 and SOX10 in mediating different miR‐637 phenotypes in gliomas.

Despite the novelty and extent of this study, several limitations that could be addressed in future studies were noted. First, we only included 40 paired human samples in this study, which is quite a limited number and thus future studies are required on circEPHB4 in a larger number of clinical samples.

Secondly, although bioinformatic analysis provided miR‐637 and SOX10 as important clues for this study, it is important to apply a systemic approach to profile miRNA expressions in glioma cells with altered expression of circEPHB4, which will help to identify other miRNA important for circEPHB4 and also for the pathogenesis of gliomas. Similarly, systematically exploring the potential targets of miR‐637 will also improve our understanding of glioma development. Also, although analysis of TCGA dataset revealed a significant correlation of higher SOX10 expression with the reduced overall survival (3 and 5 years) of glioma patients, and the median survival for patients with high SOX10 expression was shorter than that for patients with low SOX10 expression, other *in silico* validation about circEPHB4 and miR‐637 from public data is needed.

Thirdly, we chose to focus on SHG‐44 and LN229 cells, and not A172 cells in this study, mainly because the endogenous circEPHB4 level was higher in the former two cells than in A172 cells. Considering that the up‐regulated circEPHB4 and SOX10 and the reduced miR‐637 were also detected in A172 cells, when compared with normal NHA cells, we speculate that the circEPHB4/miR‐637/SOX10 axis may also act in A172 cells; this awaits further verification in future studies.

Fourthly, this is the first study demonstrating the impact of circEPHB4 on glycolysis; the significance of glycolysis and metabolic reprogramming in gliomas justifies the dedication of future studies to understand the detailed underlying mechanisms.

Fifthly, we used subcutaneous xenograft model for the *in vivo* analysis, which provided minimal information on the crosstalk between gliomas and its microenvironment that is known to significantly impact glioma development. Therefore, it is important for future studies to include orthotopic glioma models to assess the biological relevance and significance of the circEPHB4/mir‐637/SOX10 axis.

## 5 Conclusion

In this study, we indicated that circEPHB4 stimulated the stemness properties as well as the self‐proliferation of glioma cells by sponging miR‐637, thus releasing its suppression on SOX10. We provided seminal evidence that the circEPHB4/miR‐637/SOX10 axis critically regulated glioma stemness and proliferation; effective strategies targeting this axis as potential therapy for malignant gliomas could be explored. Our study might also justify follow‐up studies to further investigate more mechanisms, such as the impact of this axis in regulating other malignancy‐related biological processes during glioma development.

## Ethics approval

This research was approved by the Ethics Committee of Xiangya Hospital, Central South University (Changsha, Hunan, China) and all participants provided written consent.

## Conflict of interest

The authors declare no conflict of interest.

## Authors’ contributions

Guarantor of the integrity of the entire study: CJ, JL. Study concepts: CJ, JL. Study design: CJ, JL, JZ. Definition of intellectual content: CJ, JL. Literature research: JL, XL, CJ. Clinical studies: JZ, ZZ, MW, JL, XL, YL, BL. Experimental studies: CJ. Data acquisition: CJ. Data analysis: CJ. Statistical analysis: CJ, MW. Manuscript preparation: CJ. Manuscript editing: CJ. Manuscript review: CJ, JL, JZ, JL.

### Peer Review

The peer review history for this article is available at https://publons.com/publon/10.1002/1878‐0261.12830.

## Supporting information


**Fig S1.** SOX10 protein levels were higher in glioma tissues than in normal tissues.

**File S1.** Plasmid maps of overexpressing circEPHB4 (hsa_circ_0081519), miR‐637 and SOX10, respectively.

**File S2.** Sequences of human circEPHB4 (hsa_circ_0081519), miR‐637 and SOX10 and the shRNA sequences targeting each of these three molecules.
